The article "Opa1 Reduces Hypoxia-Induced Cardiomyocyte Death by Improving Mitochondrial Quality Control" was retracted in 2022. Reasons: original data or images not available; unreliable data; concerns about the data.

# Opa1 Reduces Hypoxia-Induced Cardiomyocyte Death by Improving Mitochondrial Quality Control

**DOI:** 10.3389/fcell.2020.00853

**Published:** 2020-08-28

**Authors:** Ting Xin, Wei Lv, Dongmei Liu, Yongle Jing, Fang Hu

**Affiliations:** Department of Cardiology, Tianjin First Center Hospital, Tianjin, China

**Keywords:** post-infarction cardiac injury, Opa1, mitochondrial quality control, mitochondria, hypoxia

## Abstract

Mitochondrial dysfunction contributes to cardiovascular disorders, especially post-infarction cardiac injury, through incompletely characterized mechanisms. Among the latter, increasing evidence points to alterations in mitochondrial quality control, a range of adaptive responses regulating mitochondrial morphology and function. Optic atrophy 1 (Opa1) is a mitochondrial inner membrane GTPase known to promote mitochondrial fusion. In this study, hypoxia-mediated cardiomyocyte damage was induced to mimic post-infarction cardiac injury *in vitro*. Loss- and gain-of-function assays were then performed to evaluate the impact of Opa1 expression on mitochondrial quality control and cardiomyocyte survival and function. Hypoxic stress reduced cardiomyocyte viability, impaired contractile/relaxation functions, and augmented the synthesis of pro-inflammatory mediators. These effects were exacerbated by Opa1 knockdown, and significantly attenuated by Opa1 overexpression. Mitochondrial quality control was disturbed by hypoxia, as reflected by multiple mitochondrial deficits; i.e., increased fission, defective fusion, impaired mitophagy, decreased biogenesis, increased oxidative stress, and blunted respiration. By contrast, overexpression of Opa1 normalized mitochondrial quality control and sustained cardiomyocyte function. We also found that ERK, AMPK, and YAP signaling can regulate Opa1 expression. These results identify Opa1 as a novel regulator of mitochondrial quality control and highlight a key role for Opa1 in protecting cardiomyocytes against post-infarction cardiac injury.

## Introduction

Acute myocardial infarction (AMI) is a common complication of ischemic cardiomyopathy, a major cause of morbidity and mortality worldwide (Davidson et al., 2018; Heusch, 2018). AMI leads to cardiomyocyte death through either apoptosis or necrosis, with subsequent impairment of cardiac activity (Chaudhuri et al., 2020). Unlike skeletal muscle cells, cardiomyocytes have a limited capacity for regeneration or proliferation. The damaged myocardium activates several mechanisms to sustain cardiac function, including an inflammatory response to remove injured cells, stimulation of fibroblast to repair infarcted tissue, augmentation of angiogenesis to enhance blood supply, and activation of neurohumoral mechanisms to maintain cardiac output (Zhou et al., 2018b; Harhous et al., 2019; Song and Li, 2019). However, dysregulation of these compensatory mechanisms induces adverse cardiac remodeling, a series of maladaptive events leading to post-infarction myocardial injury (Santin et al., 2020). Although chronic hypoxic stress has been identified as a key pathological alteration in the post-infarcted heart, the molecular mechanisms underlying hypoxia-induced myocardial injury remain little understood (Choong et al., 2019).

Cardiomyocytes require a constant supply of oxygen to generate ATP through tight coupling of the tricarboxylic acid cycle and oxidative phosphorylation in mitochondria. Accordingly, decreased oxygenation following AMI impairs cardiomyocyte metabolism and triggers hypoxic damage (Wu L. et al., 2019; Zeng and Chen, 2019). These effects are largely mediated by mitochondrial dysfunction, which leads to oxidative stress and activation of cell death programs (Zhou et al., 2017; Yuan et al., 2019; Zhang et al., 2019b). In view of the therapeutic relevance of sustaining mitochondrial function during post-infarction cardiac injury, extensive research has focused on understanding the mechanisms that govern mitochondrial dynamics (Wang and Song, 2018; Liu et al., 2019). In particular, significant efforts have been recently undertaken to identify and manipulate key components of the mitochondrial quality control system regulating mitochondrial turnover and function (Qiu et al., 2019; Thai et al., 2019; Wang et al., 2020b,c,d). Still, significant gaps remain in our understanding of the alterations in the mitochondrial quality control machinery occurring during post-infarction cardiac injury.

Our previous study reported a novel function afforded by optic atrophy 1 (Opa1), a mitochondrial inner membrane GTPase, in protecting cardiomyocytes against chronic hypoxic stress (Xin and Lu, 2020). Specifically, we showed that increased Opa1 expression stimulated mitophagy and inhibited mitochondrial oxidative stress, effectively attenuating hypoxia-mediated cardiomyocyte apoptosis (Xin and Lu, 2020). In light of these findings, and based on available evidence indicating the involvement of Opa1 in the regulation of multiple aspects of mitochondrial dynamics, i.e., mitophagy (Zhang et al., 2019a), fission and fusion (Chen et al., 2020; Elshaarawy et al., 2020), oxidative stress (Yang et al., 2020), metabolism (Schuler and Hughes, 2020), and apoptosis (Zhang et al., 2019a), the present work investigated whether Opa1 expression protects cardiomyocytes against apoptosis mediated by hypoxic stress by restoring mitochondrial quality control mechanisms.

## Materials and Methods

### Primary Cardiomyocyte Culture

Normal mouse cardiomyocytes were isolated from 1-day-old C57BL/6 mice (Wang et al., 2020a). Heart ventricles were cut and minced into 1 mm^3^ pieces and digested with 0.2% collagenase II for 2 h on ice. Digested tissues were pipetted and strained with a 70 μm strainer. Cells were collected and cultured with DMEM supplemented with 10% FBS (Invitrogen, Carlsbad, CA, United States). To mimic post-infarction cardiac injury *in vitro*, hypoxia was induced by culturing cells at 37°C in a 5% CO_2_, 95% N_2_ atmosphere for 24 h (Xin and Lu, 2020). To inhibit the MAPK/ERK, MAKPK/JNK, MAPK/p38, AMPK, Hippo/MST1 and Hippo/YAP pathways, the following blockers were respectively used: SB203580 (2 μM for 2 h), SP600125 (5 mM for 3 h), SCH772984 (5 μM for 2 h), Compound C (3 nM for 5 h), XMU-MP1 (2 nM for 6 h), and verteporfin (3 mM for 3 h). All these inhibitors were purchased from Selleck Chemicals, Houston, TX, United States.

### siRNA Transfection

Cells were transfected with 50 nM Opa1 siRNA or control (scrambled) siRNA (Santa Cruz Biotechnology, Inc., Santa Cruz, CA, United States) in serum-free, antibiotic-free DMEM containing 4 μL of siRNA transfection reagent (Santa Cruz Biotechnology, Inc.). After 6 h, the medium was replaced with fresh medium containing 10% FBS (Lionnard et al., 2019). The cells were then cultured for 48 h before downstream experiments.

### Adenovirus Construction and Transfection

Recombinant Opa1-expressing adenoviruses were constructed by Genechem (Shanghai, China). Cells were infected with purified Opa1-expressing adenoviruses or with adenoviruses containing empty plasmids (control) for 24 h at a multiplicity of infection (MOI) of 50. The medium was then replaced with fresh medium (Wolint et al., 2019) and successful infection was confirmed through western blotting.

### Ca^2+^ Transient and Contractility Measurements

The mechanical properties of ventricular myocytes were assessed through a video-based detection system as previously described (Zhou et al., 2018c). In brief, a laminin-coated coverslip with cells attached was placed in a chamber mounted on the stage of an inverted microscope (Motic AE31) and perfused (about 1 mL/min at 37°C) with Tyrode’s buffer. Cardiomyocytes were stimulated to contract at 0.5 Hz (Matthews et al., 2019). Changes in sarcomere length during shortening and relengthening were captured and analyzed using SoftEdge^TM^ software (IonOptix, Westwood, MA, United States). To evaluate Ca^2+^ transients, cardiomyocytes were loaded with 0.5 μmol/L Fura2-AM (Life Technologies, Carlsbad, CA, United States), a Ca^2+^-sensitive indicator, for 10 min at 37°C. IonOptix was used to record fluorescence emission and to simultaneously perform contractility measurements (Morton et al., 2019).

### Reactive Oxygen Species Measurement

Cellular ROS generation was detected as described previously (Kohlhauer et al., 2019). In brief, cells grown at specified culture conditions on 24-well or 6-well plates were incubated with 2.5 μM dihydroethidium (DHE, Beyotime, Shanghai, China) for 30 min. The medium was then replaced and cells incubated for another 30 min. ROS generation was assessed by fluorescence microscopy.

### ATP Measurement

Cellular ATP levels were measured using an ATP Assay Kit (Abcam, #ab83355) according to manufacturer’s instructions (Li S. et al., 2019). Briefly, 20 mg of sample was homogenized on ice using a hand-held homogenizer in ice-cold 2M perchloric acid (PCA). Homogenates were then incubated on ice for 45 min before centrifugation at 13,000 g for 2 min at 4°C. Supernatants were collected, and PCA neutralized with ice-cold 2M KOH. Sample pH was adjusted between 6.5 and 8.0 as needed. Samples were then 10 centrifugated again at 13,000 g for 2 min at 4°C and used for the colorimetric assay (Aalto et al., 2019).

### ELISA

Secreted IL-8, TNF-α, and MMP9 levels were measured using ELISA kits (Wuhan USCN Business Co., Ltd., Wuhan, China). Following experimental treatments, cell culture media were obtained and coagulated for 30 min. Samples were collected by centrifugation (3, 000 rpm/min for 10 min). ELISA was performed according to the manufacturer’s instructions (Araki et al., 2018). Briefly, samples were diluted at a ratio of 1:2 in the provided diluent to a final volume of 100 μL and added (in duplicate) into microtiter plates (96-well flat-bottom) for 24 h. The plates were washed three times with diluent, and monoclonal antibodies diluted 1:1000 in diluent were added to each well and incubated for 3 h at room temperature. After washing, a peroxidase-conjugated anti-rabbit antibody (diluted 1:1000) was added to each well and incubated at room temperature for 1 h. After addition of streptavidin-enzyme, substrate, and stop solution, the concentrations of IL-8, TNF-α, and MMP9 were determined by absorbance measurements at 450 nm in a spectrophotometer (Edwards et al., 2018). The standard curve demonstrated a linear relationship between optical density (OD) and test concentrations. Total protein was measured by Lowry’s method using bovine serum albumin (BSA) as a standard.

### Apoptosis Assay

Apoptosis was detected using a terminal deoxynucleotidyl transferase dUTP nick end labeling (TUNEL) assay kit (Roche Applied Science, Mannheim, Germany) (Le et al., 2019) in accordance with the manufacturer’s instructions using 4-μm thick paraffin-embedded samples (Bittremieux et al., 2019). Slices were mounted and the percentage of TUNEL positive nuclei were calculated.

### Cell Viability Assay

Cell viability was measured using the 3- [4,5-dimethylthiazol-2-yl]-2,5 diphenyltetrazolium bromide (MTT) assay. Freshly isolated cardiomyocytes were seeded into 96-well plates at a density of 1 × 10^5^ cells/well and incubated overnight. The cells were then transduced with Opa1-expressing adenovirus for 72 h. Over the last 24 h of this time period, the cells were exposed to hypoxia or kept in normoxic conditions and then incubated with MTT for 2-3 h (Jiang et al., 2019). Following addition of DMSO, absorbance was detected on a μQuant^TM^ microplate reader (Bio-Tek Instruments, United States) at 570 nm. Cell viability (%) was calculated as [Absorbance at × concentration (virus sample)]/[Absorbance at 0 concentration (control)] × 100 (Su et al., 2019; Zhou X. L. et al., 2019).

### qPCR Validation of Virus Copy Number

Cells were plated in 6-well plates at a concentration of 2 × 10^5^ cells/mL and incubated overnight. RNA was extracted from lentivirus-treated samples using TRI Reagent^®^ (Sigma, United States) and the yield and purity of RNA were then assessed using a Nanodrop instrument (Eppendorf, United States) (Hysi et al., 2019). All qPCR reactions were performed in a final volume of 20 μL reaction mixture containing 1X of iTaq universal probes reaction mix (Bio-Rad, United States), 0.5 μM of each forward and reverse primer, 0.25 μM of TaqMan probe, 1 unit of iScript reverse transcriptase, and 300 ng of RNA. No-template controls were included in each run. RNA conversion to cDNA, cDNA amplification, and quantification was performed using a Bio-Rad CFX96^TM^ Touch Real-Time PCR Detection System (Bio-Rad). Data analysis was performed using CFX Manager^TM^ Software version 1.6 (Bio-Rad Laboratories, Inc.) (Na et al., 2019).

### Western Blot Analysis

Protein aliquots (30 μg) from each sample were resuspended in sodium dodecyl sulfate-polyacrylamide gel electrophoresis (SDS-PAGE) loading buffer, boiled at 95°C for 10 min, and separated using 11.5% SDS-PAGE gels (Ham et al., 2019). Following electrotransfer to polyvinylidene fluoride membranes and blocking in 5% non-fat milk (1 h at room temperature), the membranes were incubated overnight at 4°C with an anti-Opa1 antibody (Abcam) in 1X Tris-buffered saline, 0.1% Tween^®^ 20 (TBST) with 2% bovine serum albumin (BSA). The membranes were then washed three times for 10 min with TBST and subsequently incubated with HRP-conjugated secondary antibodies at room temperature for 1 h. Following ECL detection, protein bands were visualized using an Imaging System. GAPDH was used as loading control (Peng et al., 2018).

### Statistical Analysis

SPSS 17.0 (SPSS Inc., Chicago, United States) software was used to perform statistical analysis. Differences between treatment means were assessed by one-way ANOVA. Results are presented as the mean ± standard deviation. *P* < 0.05 indicated significance. All experiments were performed at least three times.

## Results

### Overexpression of Opa1 Attenuates Cardiomyocyte Damage and Dysfunction Induced by Hypoxic Stress

To assess the role of Opa1 in post-infarction cardiac damage, an *in vitro* model was established by introducing Opa1-expressing adenoviral vectors (Ad-Opa1) or a siRNA targeting Opa1 (si-Opa1) into primary cardiomyocytes isolated from neonatal mice. Post-infarction myocardial injury was mimicked by exposing cells to 24-h hypoxia as previously described (Xin and Lu, 2020), and biomarkers related to cardiac damage were then measured in culture media through ELISA. Compared to the control group, hypoxia stress significantly upregulated troponin T (TnT), troponin I (TnI), and creative kinase MB (CK-MB) levels. Interestingly, the upregulation of these three proteins was prevented by Ad-Opa1 transduction, whereas si-Opa1 transfection further augmented TnT, TnI, and CK-MB secretion (Figures 1A–C). These data indicate that hypoxia-mediated cardiomyocyte damage is counteracted by Opa1 activity. This finding was confirmed through analyzing cardiomyocytes’ contractility and relaxation dynamics. As shown in Figures 1D,E, hypoxic stress significantly impaired maximal shortening and relengthening velocities. Opa1 overexpression not only reversed this effect, but also increased cardiomyocytes’ relaxation time. In contrast, Opa1 knockdown significantly impaired these parameters. Using immunofluorescence, we found that the expression of myosin, the primary motor protein regulating cardiomyocyte contraction, was downregulated by hypoxia. This phenomenon was more pronounced after Opa1 knockdown, and prevented by Opa1 overexpression (Figures 1F,G). These results indicate that Opa1 expression ensures cardiomyocyte function and attenuates hypoxia-related damage.

**FIGURE 1:** Overexpression of Opa1 attenuates cardiac damage and dysfunction induced by hypoxic stress. **(A–C)** ELISA analysis of troponin T (TnT), troponin I (TnI), and creatine kinase MB (CK-MB) secretion by Opa1-overexpressing (Ad-Opa1) and Opa1-knockdown (si-Opa1) cardiomyocytes subjected to 24 h hypoxia exposure. **(D,E)** Analysis of cardiomyocyte contractile properties. Maximal shortening and relengthening velocities were measured using a SoftEdge MyoCam system. **(F,G)** Myosin immunofluorescence results. ^∗^*p* < 0.05.

### Opa1 Overexpression Reduces Cardiomyocyte Inflammation and Apoptosis

Chronic hypoxic stress is associated with activation of inflammatory responses and apoptosis in the post-infarcted heart (Xie et al., 2019). To explore whether Opa1 expression influences inflammation and apoptosis in hypoxic cardiomyocytes, we analyzed the expression of pro-inflammatory mediators and evaluated apoptosis induction following Opa1 overexpression and knockdown. Results of qPCR analysis demonstrated significant upregulation of the pro-inflammatory cytokines IL-8 and TNFα, as well as of MMP9 expression, in hypoxia-treated cardiomyocytes. Suggesting a protective role for Opa-1, IL-8, TNFα, and MMP9 expression was further upregulated upon si-Opa1 transfection, and inhibited instead in cells transduced with Ad-Opa1 (Figures 2A–C). Further evidence that hypoxia-related cardiomyocyte inflammation is alleviated by Opa1 overexpression was obtained through ELISA, which showed concomitant changes in secreted IL-8, TNFα, and MMP9 levels (Figures 2D–F).

**FIGURE 2:** Opa1 reduces cardiomyocyte inflammation and apoptosis. **(A–C)** Analysis of IL-8, TNFα, and MMP9 expression through qPCR. **(D–F)** ELISA analysis of IL-8, TNF-α, and MMP-9 secretion. **(G)** MTT viability assay results. **(H,I)** Apoptosis assay results. TUNEL staining was applied to quantify the number of apoptotic cardiomyocytes following hypoxic stress. ^∗^*p* < 0.05.

To evaluate whether Opa1 confers protection against hypoxia-mediated cardiomyocyte death, viability and apoptosis were next examined by MTT and TUNEL assays. Results showed that cardiomyocyte viability was reduced (Figure 2G), while the number of TUNEL-positive cells was increased (Figures 2H,I), following hypoxic stress. Consistent with a protective role for Opa1, these effects were respectively exacerbated and counteracted by Opa1 silencing and overexpression.

### Opa1 Overexpression Activates Mitophagy and Mitochondrial Biogenesis in Hypoxia-Treated Cardiomyocytes

Considering the key role played by mitochondrial quality control in regulating cardiac function (Zhou H. et al., 2019), we next asked whether Opa1 protects cardiomyocytes against hypoxic stress through improving mitochondrial quality control. To this end, we first evaluated mitophagy and mitochondrial biogenesis. Results of qPCR analysis demonstrated significant upregulation of the mitophagy markers ATG5, Parkin, and Beclin1 following hypoxia (Figures 3A–C). Suggesting that mitophagy activation requires Opa1, this effect was enhanced by Opa1 overexpression and suppressed by Opa1 knockdown. These findings were further confirmed using mt-Keima, a mitochondrial targeted, pH-sensitive fluorescent fusion protein that shows a shift in fluorescence when damaged mitochondria are incorporated into lysosomes during mitophagy. As shown in Figures 3D,E, mitophagy was significantly increased after exposure to hypoxia, further enhanced by Opa1 overexpression, and reduced instead after Opa1 knockdown.

**FIGURE 3:** Opa1 activates mitophagy and mitochondrial biogenesis in hypoxia-treated cardiomyocytes. **(A–C)** Analysis of ATG5, Parkin, and Beclin1 expression through qPCR. **(D,E)** Mitophagy analysis in living cardiomyocytes by mt-Keima reporter assay. **(F,G)** Analysis of Tfam and PGC1α expression through qPCR. ^∗^*p* < 0.05.

Following mitophagy activation, stimulation of mitochondrial biogenesis is required to maintain cellular energy levels. Reduced mitochondrial biogenesis, evidenced by decreased transcription of *Tfam* and *PGC1*α, two markers of mitochondrial DNA synthesis, was observed in cardiomyocytes exposed to hypoxia. In turn, upregulation of *Tfam* and *PGC1*α levels in hypoxia-treated, Ad-Opa1-transduced cells indicated that mitochondrial biogenesis is enhanced by Opa1 expression (Figures 3F,G).

### Opa1 Inhibits Mitochondrial Fission and Enhances Mitochondrial Fusion

Proper functioning of the mitochondrial quality control system is not only essential for coordinated mitophagy and biogenesis, but also for the regulation of mitochondrial fission and fusion, redox balance, and bioenergetics (Tahrir et al., 2019). Therefore, we conducted a series of experiments to evaluate whether Opa1 expression in cardiomyocytes influences these latter aspects of mitochondrial dynamics under hypoxic conditions. Following 24-h hypoxia, gene expression analysis revealed upregulation of the mitochondrial fission-related genes Drp1, Mff, and Fis1 and downregulation of the mitochondrial fusion-related genes Mfn1 and Mfn2. These expression patterns were more pronounced after Opa1 knockdown, and markedly repressed by Opa1 overexpression (Figures 4A–E). These findings were further supported by mitochondrial immunofluorescence studies using Tom-20 antibody. As shown in Figures 4F,G, characteristic, spindle-shaped mitochondria were observed under normoxic conditions. After exposure to hypoxia, however, the number of spindle-shaped mitochondria was reduced whereas the percentage of small, round mitochondria was increased. Since Opa1 overexpression largely restored the ratio of spindle-shaped to round mitochondria in hypoxic cardiomyocytes, we conclude that Opa1 activity counteracts hypoxia-induced mitochondrial fission.

**FIGURE 4:** Opa1 inhibits mitochondrial fission and enhances mitochondrial fusion. **(A–E)** Analysis of Drp1, Mff, Fis1, Mfn2, and Mfn1 expression through qPCR. **(F,G)** Analysis of mitochondrial morphology using immunofluorescence. The ratio of spindle-shaped to round mitochondria was estimated. ^∗^*p* < 0.05.

### Opa1 Expression Attenuates Oxidative Stress and Increases Mitochondrial Respiration in Hypoxia-Treated Cardiomyocytes

To investigate the influence of Opa1 on mitochondrial redox balance and bioenergetics, we first assessed ROS generation in cardiomyocytes loaded with the redox-sensitive dye DHE. Indicative of oxidative stress, DHE fluorescence was increased by hypoxia. This increase was exacerbated by Opa1 knockdown and effectively neutralized following Opa1 overexpression (Figures 5A,B). Meanwhile, ELISA analysis of cell culture supernatants/cell extracts showed that the content of mitochondrial antioxidant enzymes, i.e., manganese superoxide dismutase (MnSOD), glutathione reductase (GR), thioredoxin reductase (TrxR), and peroxiredoxin (PRx), decreased rapidly in response to hypoxia (Figures 5C–F). Suggesting a protective role for Opa1 against oxidative stress triggered by hypoxia, the referred changes were more obvious in cardiomyocytes transfected with si-Opa1, but prevented by Opa1 overexpression.

**FIGURE 5:** Opa1 overexpression attenuates oxidative stress and improves mitochondrial respiration in hypoxia-treated cardiomyocytes. **(A,B)** Analysis of mitochondrial ROS production by DHE staining. **(C–F)** ELISA analysis of manganese superoxide dismutase (MnSOD), glutathione reductase (GR), thioredoxin reductase (TrxR), and peroxiredoxin (PRx) levels in (culture media from) hypoxia-treated cardiomyocytes. **(G)** Determination of mitochondrial oxygen consumption rate (OCR). **(H)** Measurement of ATP production in cardiomyocytes subjected to hypoxic stress. **(I,J)** ELISA/Colorimetric analysis of mitochondrial respiratory complex I and III activities in hypoxia-treated cardiomyocytes. ^∗^*p* < 0.05.

A key function of the mitochondrial quality control machinery is the regulation of mitochondrial bioenergetics, which is essential to sustain cardiomyocyte metabolism (Aluja et al., 2019). As shown in Figures 5G,H, hypoxia reduced both oxygen consumption rate (OCR) and ATP production in cultured cardiomyocytes, and these changes were attenuated/prevented by Opa1 overexpression. Consistent with these findings, the activity of the mitochondrial respiratory complexes I and III was downregulated by hypoxia, and this effect was also prevented by Ad-Opa1 transduction (Figures 5I,J). These results indicate that Opa1 expression helps maintain mitochondrial redox status and bioenergetic function in hypoxic cardiomyocytes.

### Opa1 Expression Is Regulated by ERK, AMPK, and YAP Signaling Pathways

The above data established the important role of Opa1 in preserving mitochondrial quality control during hypoxic stress in cardiomyocytes. However, the specific signaling pathways implicated in the regulation of Opa1 expression during hypoxia have not yet been properly defined. Based on recent studies (Zhang et al., 2016; Kashihara and Sadoshima, 2019; Ma and Liu, 2019), we analyzed whether activation of six major pathways associated to hypoxic stress in cardiomyocytes, i.e., MAPK/ERK, MAKPK/JNK, MAPK/p38, AMPK, Hippo/MST1, and Hippo/YAP, influences Opa1 transcription. As shown in Figures 6A–F, pharmacological inhibition of ERK, AMPK, or YAP, but not JNK, p38, or MST1, partly reduced Opa1 transcription in cardiomyocytes under normoxic conditions. These data indicate that Opa1 stabilization in cardiomyocytes is controlled by ERK, AMPK, and YAP activities.

**FIGURE 6:** Opa1 expression is regulated by ERK, AMPK, and YAP signaling. **(A–F)** Analysis of Opa1 expression by qPCR following pharmacological inhibition of MAPK/ERK, MAKPK/JNK, MAPK/p38, AMPK, Hippo/MST1, or Hippo/YAP. See “Materials and Methods” for details. ^∗^*p* < 0.05.

## Discussion

Over the past decade, substantial attention has been paid to the molecular mechanisms involved in acute cardiovascular damage mediated by myocardial infarction and ischemia-reperfusion injury (Dassanayaka et al., 2019; Eiringhaus et al., 2019). In contrast, much less effort has been devoted to investigating the cellular alterations underlying chronic cardiovascular disorders such as chronic heart failure and post-infarction cardiac injury. In this study, mouse neonatal cardiomyocytes were subjected to hypoxic stress to model post-infarction cardiac injury *in vitro*. Through molecular imaging and gene and protein expression analyses, we characterized several deficits in mitochondrial turnover and function that indicate that dysregulated mitochondrial quality control contributes to cardiomyocyte damage and death during hypoxia. More importantly, we identified Opa1 as a key regulator of mitochondrial quality control, which leads us to suggest that induction of Opa1 expression might be an effective means to support cardiac function under hypoxic stress conditions. As far as we known, this is the first study to explore the influence of Opa1 on mitochondrial quality control in the setting of post-infarction cardiac injury.

Myocardial infarction is most commonly caused by atherosclerosis leading to coronary artery occlusion, and determines ischemic damage of the myocardium (Hadebe et al., 2018; Heusch, 2019). Consequently, the infarcted area is invaded by inflammatory cells and fibroblasts, which mediate tissue repair and reconstruction (Botker et al., 2018; Jung et al., 2018). However, both unresolved inflammation and excessive fibrosis can potentiate post-infarction cardiac injury through mechanisms that remain incompletely understood. In the present study, we showed that hypoxic stress lasting 24 h decreased proliferation and stimulated apoptosis in primary cultures of mouse cardiomyocytes. Paralleling a decrease in myosin expression, cardiomyocytes’ contractile and relaxation functions were also impaired by hypoxic stress. Interestingly, our data also illustrated that hypoxia treatment upregulated the synthesis of pro-inflammatory (TNF-α and IL-8) and pro-fibrotic (MMP-9) factors in cultured cardiomyocytes, which corroborates and expands previous findings on the role of hypoxia as an activator of the inflammation response in the myocardium [REF]. However, the relationship between hypoxia and inflammation, as well as their combined effects on post-infarction cardiac injury, have not been completely elucidated.

Cardiomyocytes contain abundant mitochondria to generate ATP for cell metabolism and contraction. Accordingly, dysregulated mitochondrial function is linked to a variety of cardiovascular disorders such as acute ischemia-reperfusion injury, diabetic cardiomyopathy, sepsis-related myocardial depression, and heart failure (Jin et al., 2018; Zhou et al., 2018a,d). Indeed, mitochondrial damage, caused by either hypoxia and/or inflammation, is also noted in the progression of post-infarction cardiac injury (Wang and Song, 2018; Liu et al., 2019). This phenomenon was also confirmed in our present study. Furthermore, our data suggested that dysregulated mitochondrial quality control is intimately associated with mitochondrial dysfunction in hypoxic cardiomyocytes. Mitochondrial quality control comprises a range of adaptive responses that are activated by various stresses in virtually all cell types to reduce or prevent mitochondrial damage (Zhou et al., 2018e; Li et al., 2020). In the present study, disrupted mitochondrial quality control following hypoxic stress was evidenced by multiple alterations in mitochondrial morphology and function, namely increased fission, defective fusion, decreased biogenesis, increased oxidative stress, and blunted respiration. Suggesting a key regulatory role for Opa1 on mitochondrial quality control, overexpression of Opa1 normalized mitochondrial fission/fusion dynamics, promoted mitochondrial biogenesis, neutralized mitochondrial oxidative stress, and improved mitochondrial respiration in hypoxic cardiomyocytes. Of note, although our study identified Opa1 as a potential target for the treatment of post-infarction cardiac injury, there are yet no effective drugs to enhance Opa1 expression.

Our results are in agreement with previous studies showing that Opa1 activity exerts beneficial effects during cardiac injury by reducing reperfusion-mediated cardiomyocyte damage through upregulation of mitochondrial metabolism (Luo et al., 2019) and promotion of mitochondrial fusion (Zhang et al., 2019a). Reflecting also the essential role of Opa1 in cellular energy homeostasis, previous studies in mouse models of skeletal muscle atrophy [51], prion disease [52], and liver dysfunction (Li L. et al., 2019; Wu W. et al., 2019; Lee et al., 2020) showed that Opa1 protects myocytes, neurons, and hepatocytes by improving mitophagic flux and mitochondrial dynamics and metabolism.

There are some limitations in the present study. First, although we identified ERK, AMPK, and YAP kinases as transcriptional modulators of Opa1 expression, further molecular assays are needed to clarify the mechanisms mediating downregulation of Opa1 expression in hypoxic conditions. Second, since post-infarction cardiac injury is also associated with endoplasmic reticulum stress, unfolded protein response, and abnormal intracellular calcium signaling (Zhu et al., 2018; Zhang et al., 2020), more studies are required to explore the influence of mitochondrial quality control on these pathological alterations. Third, to confirm the therapeutic relevance of the present findings, our *in vitro* results need to be validated in animal models of post-infarction cardiac injury.

In summary, our research indicates that upregulation of Opa1 expression prevents cardiomyocyte apoptosis and sustains cardiomyocyte function during hypoxic stress by enhancing mitochondrial turnover and respiratory capacity. These findings provide novel insight into the pathogenesis of post-infarction cardiac injury and suggest that therapies aimed at stimulating Opa1 expression may be valuable to attenuate the sequelae of this common health condition.

## Data Availability Statement

All datasets generated for this study are included in the article/supplementary material.

## Ethics Statement

The animal study was reviewed and approved by the Tianjin First Central Hospital.

## Author Contributions

TX and FH designed and performed the parts of experiments. WL and DL collected all the data and prepared the figures. YJ and TX wrote the manuscript. All authors approved this submission.

## Conflict of Interest

The authors declare that the research was conducted in the absence of any commercial or financial relationships that could be construed as a potential conflict of interest.
